# Mutation Profile Assessed by Next-Generation Sequencing (NGS) of Circulating Tumor DNA (ctDNA) in Chinese Lung Adenocarcinoma Patients: Analysis of Real-World Data

**DOI:** 10.1155/2021/8817898

**Published:** 2021-05-04

**Authors:** Songchen Zhao, Xiaofeng Cong, Ziling Liu

**Affiliations:** The First Hospital of Jilin University, China

## Abstract

**Background:**

Genomic testing gives guidance to the treatment options in lung adenocarcinoma patients, but some patients are unable to obtain tissue samples due to lesion location or intolerance. Cell-free circulating tumor DNA (ctDNA) tested in plasma or pleural effusion is an advanced access to solve the problem. Our study descriptively identified the genetic variations of advanced Chinese lung adenocarcinoma patients and analyzed the overall survival of patients with EGFR mutations.

**Methods:**

A total of 152 patients' plasma samples were included, and gene mutations were detected by NGS using an Illumina Miseq tabletop sequencer.

**Results:**

Frequencies of altered were EGFR 46.05%, ALK 7.24%, KRAS 6.58%, PIK3CA 6.58%, PTEN 2.63%, HER2 1.97%, MET 1.97%, BRAF 1.32%, NF1 1.32%, and ROS1 0.66%. We identified 48 cases with double or triple driver gene mutations. Multiple mutations were more frequently observed in EGFR and PIK3CA genes. Patients harboring coexistent mutations with an EGFR mutation tended to have a shorter overall survival than those with exclusively EGFR mutations.

**Conclusion:**

EGFR, ALK, and KRAS were common driver gene in Chinese patients with stage IV lung adenocarcinoma. Multiple mutations were detected in the ctDNA samples and involve more EGFR and PIK3CA mutations. The existence of coexisting gene mutations may have adverse effects on the prognosis of patients with EGFR mutation. The unknown mutations discovered by NGS may provide new targets for gene targeting therapy, and ctDNA test by NGS is an effective method for making appropriate treatment choices.

## 1. Introduction

At present, lung cancer is still the leading cause of cancer incidence and mortality worldwide [1]. However, the mortality of lung cancer has dropped in the last decade which is related to the development of targeted therapies and other advanced therapies [2]. Targeted molecular therapy has improved the outcomes of patients with advanced nonsmall cell lung cancer (NSCLC) who harbor sensitive mutations [3, 4]. Therefore, genomic testing is crucial to explore potential molecular targets for the treatment of lung cancer, thereby reducing the mortality of NSCLC. The National Comprehensive Cancer Network treatment guidelines advocate actionable mutation screening as standard of care, and genomic retesting is necessary at a time of tumor progression [5]. However, tissue samples are often difficult to obtain due to lesion location or intolerance, especially in relapsed and metastatic settings. Liquid biopsy is a noninvasive, clinically actionable, and reliable method to solve the problem. NGS uses ctDNA shed from tumors into the circulation as a substrate for mutation detection. Recent studies showed that plasma NGS testing demonstrates a marked increase of the detection of therapeutically targetable mutations [6, 7]. Furthermore, the detection of ctDNA by NGS allows huge amounts of variants to be identified in each sample on a single platform. In our study, we identified the genomic mutation profile of ctDNA in real-world Chinese stage IV lung adenocarcinoma patients using the NGS panel.

## 2. Methods

### 2.1. Patients

A total of 152 patients who were pathologically diagnosed with stage IV lung adenocarcinoma were included in our study. These eligible patients received NGS assays in The First Hospital of Jilin University from January 2016 to December 2019. 14 genes (EGFR, ALK, KRAS, PIK3CA, PTEN, HER2, MET, BRAF, AKT1, NF1, ROS1, RET, NRAS, and MAP2K1) were detected for 94 patients, 139 genes were detected for 25 patients and 425 genes for 33 patients, and the choices were made by patients and their physicians.

### 2.2. Blood Samples and ctDNA Extraction

5 ml of whole blood was collected by ethylenediamine tetraacetic acid (EDTA) blood collection tubes then transported at ambient temperature to Nanjing Shihe Jiyin Biotech Inc. (Nanjing, China) no more than 72 h. Blood was centrifuged at 1800 × g for 10 minutes at 4°C to remove blood cells. Then, the supernatant was centrifuged at 16000 × g for 10 minutes at 4°C to remove any remaining cells. Circulating tumor DNA was extracted from 2 ml plasma, by digestion in 100 *μ*l proteinase K buffer for 10 min at 37°C followed by purification with the NucleoSpin Plasma XS kit with modified protocols. The purified ctDNA is quantified by a Picogreen fluorescence assay using the provided lambda DNA standards (Thermo Fisher Scientific, Waltham, MA, USA).

### 2.3. ctDNA Sequencing and Analysis

The 5′-biotinylated probe solution is provided as capture probes, and the baits target cancer-related genes. Hybridization, target amplifcation, barcode library preparation, and size selection were performed according to the manufacturer's protocols. After amplification, the samples are purified by AMPure XP beads, quantified by qPCR (Kapa Biosystems, Boston, USA), and sized on bioanalyzer 2100 (Agilent Technologies, China). Libraries are normalized to 2.5 nM and pooled. Deep sequencing is performed on Illumina HiSeq 4000 using PE75 V1 Kit. Cluster generation and sequencing are performed according to the manufacturer's protocol.

Base calling was performed using bcl2fastq (Illumina, Inc. San Diego, California, USA) to generate sequence reads in FASTQ format (Illumina, Inc. San Diego, California, USA). Quality control was applied with Trimmomatic [8]. High-quality reads were mapped to Human Genome Build 19 (Hg19)/GRCh 37 reference sequence. Single nucleotide variants and short insertions/deletions were identified using VarScan2 [9], and copy number variations (CNVs) were identified using ADTEx [10]. All the above experimental steps were carried out by Nanjing Shihe Jiyin Biotech Inc. (Nanjing, China).

### 2.4. Data Collection and Statistics

Demographic characteristics of the patients were collected from the medical records from The First Hospital of Jilin University. Patients that harbored EGFR mutations were treated with EGFR-TKIs for first-line treatment while the others with chemotherapy. Overall survival (OS) was defined as the time from the molecular analysis assessment date to the date of death or final follow-up (2021.01.09). Survival curves were estimated by the Kaplan-Meier method for the patients with EGFR mutations. The relationship between mutation status and patient characteristics was compared by using the chi-square test for qualitative variables or a nonparametric test for quantitative variables. All data were analyzed by SPSS version 25.0 (IBM Corporation, Armonk, NY, USA), *p* < 0.05 was considered to be statistically significant.

## 3. Results

### 3.1. Patient Characteristics and Gene Mutation Patterns

152 patients with stage IV lung adenocarcinoma were included in this study. The cohort included 80 male patients and 72 female patients; 86 were over 60 years old and 66 under 60 years old (Table 1). With regard to the 14 genes tested in all patients, 109 patients (71.7%) harbored at least one genomic mutation. Frequency of altered was EGFR 46.05%, ALK 7.24%, KRAS 6.58%, PIK3CA 6.58%, PTEN 2.63%, HER2 1.97%, MET 1.97%, BRAF 1.32%, NF1 1.32%, and ROS1 0.66% (Figure 1). The EGFR mutation was more common in females, <60 years, but in our cohort, these differences were not statistically significant (*p* > 0.05) (Table 1). There was no difference among EGFR (-) vs. exclusively EGFR mutated cases vs. EGFR +coexistent mutations with sex and age (Table 2).

### 3.2. Distribution of Common Gene Mutations

EGFR mutations were detected in 70 patents of the total 152 patients, including 34 who harbored double or triple EGFR gene mutations. The most common EGFR mutations were exon-19 deletions (51.72%, 15/29), followed by L858R (34.48%, 10/29) in patients who harbored single mutation (Table 3). 17 patients with tumor recurrence harbored T790M mutation, and we also found one untreated patient detected with T790M mutation. In addition, insert mutation of exon-19, exon-20, L861Q mutation, and copy number amplification was detected in 1 case each. EML-4/ALK fusion (8/11) was the most common mutation in the ALK gene. The remaining of these is located in exon-19 or exon-20. PIK3CA mutations were detected in 10 patients, most of those located on E545K in exon-9(6/10), and the others in exon-20. KRAS mutations were identified in 10 patients, and all of them were on exon-2. G12C (5/10) was the most frequent mutation detected in the KRAS gene. PTEN mutations were detected in 6 patients, 1 of them was truncation mutation, and the others were point mutations. HER2 mutations: insertion mutation in exon-20 (2 cases) and germ line mutation (1 case) were identified in 3 cases. BRAF mutations were identified in 2 patients; all of them were V600E mutation. 2 cases of NF1 mutations and 1 case of ROS1 fusion mutation were also detected. The specific distribution was shown in Table 4.

### 3.3. Multiple and Unknown Gene Mutations Detected in ctDNA of Stage IV Lung Adenocarcinoma

Out of 109 patients with genetic variations, 43 patients were found to harbor multiple mutations (29 exclusively EGFR mutations and 14 coexisting mutations). Of the exclusively double or triple EGFR mutations, most were EGFR sensitive mutation (exon − 19 deletion/exon − 21 L858R) + T790M (11/34), followed by exon − 19 deletion + gene copy number amplification (3/34). Coexistent mutations were detected in 14 patients: 4 EGFR+PIK3CA, 1 EGFR+PIK3CA + PTEN, 3 EGFR + PTEN, 1 EGFR+HER2, 1 EGFR+KRAS, 1 PIK3CA + HER2, 1 PIK3CA + KRAS, 1EGFR + NF1, and 1 EGFR + MET (Table 5); in this small cohort, EGFR remains the most common mutation gene (12/14) followed by PIK3CA (7/14). We also detected 13 patients with gene mutations whose functions were still unclear (Table 6).

### 3.4. Overall Outcome in Patients Harboring EGFR Mutations

Out of 70 patients harboring EGFR mutations, 58 were exclusively EGFR mutations (29 single EGFR mutations and 29 double or triple EGFR mutations), and 12 were coexistent mutations. All of these patients received TKI therapy as first line treatment. After the exclusion of 11 patients who were lost to follow-up, survival data were obtained in 59 patients. Patients harboring coexistent mutations with an EGFR mutation tended to experience worse prognosis than those with exclusively EGFR mutations (OS = 21.0 vs. 16.0 months, *p* = 0.104, Figure 2) although not statistically significant.

## 4. Discussion

We tested 152 Chinese stage IV lung adenocarcinoma liquid samples to analysis gene mutation patterns by NGS. High throughput, multiplex tests implementable for clinical are necessary to direct therapy choice for individual patients. Several studies have demonstrated that NGS is a capable method, which is quick, stable, and cost-effective [11–14]. Furthermore, NGS provided both the advantage of low input DNA concentration and the detection of low-frequency variants [12]. Therapies matched to ctDNA mutations monitoring during treatments demonstrated appreciable therapeutic efficacy [15].

Previous studies showed that the most common EGFR mutations in NSCLC were exon-19 deletions and point mutation L858R in exon-21, which were referred to as sensitive mutations and benefited from RGFR-TKIs' therapy [16]. We conducted genomic test in 152 Chinese patients; in our cohort, the EGFR sensitive mutation rate was significantly higher than those declared in American patients with lung adenocarcinomas (46.05% vs. 19.0%) [17]. It shows that ethnic difference exists in the distribution of gene mutations. As EGFR sensitive mutations were more likely to occur in lung adenocarcinoma [16], our incidence was higher than previously reported Chinese NSCLC patients (46.05% vs. 34.8%) [18]. We detected a case of L681Q mutation on exon-21 which was considered very rare. Patients with L681Q mutations showed poor outcomes compared with those who harbored sensitive mutations [19, 20]. Inspiringly, several clinical trials have demonstrated that afatinib was active in patients' harbored L681Q mutation [21, 22]. T790M mutation was always acquired in lung adenocarcinoma patients after exposure to EGFR-TKIs' therapies, which related to resistance to the first or second generation of TKIs [23]. In our study, 21 patients with T790M mutations were identified including a case without TKI therapy history. EGFR gene mutations were observed commonly in female, <60 years, and adenocarcinoma patients with NSCLC in previous reports [18]. In our cohort, EGFR mutation was not significantly correlated with age and gender. Our small sample size and fixed pathologic type may result to the inconsistent. And the *p* value is near 0.05 for gender difference, which may be due to the limited sample sizes. In our cohort, the mutation status of EGFR was not associated with age (*p* > 0.05) (Table 2). EGFR negative and EGFR + coexistent mutations appear to be more common in females, whereas exclusively EGFR-mutated cases were more likely to occur in males (Table 2), but the differences were not statistically significant.

The incidence of ALK gene fusion mutation was about 3.8% in the Asian lung adenocarcinoma population [24]. In our cohort, 9 of 152 patients with stage IV lung adenocarcinoma had positive ALK gene fusion mutations, with a mutation rate of 7.24%, slightly higher than the reported level. Almost all the ALK gene fusion mutations detected were EML4-ALK fusion mutations (8/11). 2 cases of unknown point mutations (D1311E, K1101N) on the ALK gene were detected, whose function was still unclear in the development of tumor.

The incidence of KRAS gene mutation was 15%-25% in patients with nonsmall cell lung cancer [25]. In our cohort, 10 cases with KRAS gene mutation were detected in 152 patients with stage IV lung adenocarcinoma, with a mutation rate of 6.58%, slightly lower than the reported level. Most KRAS gene mutations detected were on codon 12 of exon 2 [26, 27], which was associated with a poor prognosis and resistance to TKI therapies.

The incidence of PIK3CA gene mutation in nonsmall cell lung cancer is 2%-5% [18, 28, 29]. In 152 patients with stage IV lung adenocarcinoma, 10 were detected with PIK3CA mutations (6.58%). Most mutations occurred in exon 9 or 20 (6/4), and 7 cases of PIK3CA mutations coexisted with other drive genes at the same time: 5 PiK3CA + EGFR, 1 PIK3CA + HER2, and 1 PIK3CA+ KRAS. In our cohort, PIK3CA mutations tended to accompany other driver genes such as EGFR and KRAS coexist and always occur on exon 9 or 20, and these results showed consistency with a previous study [29].

In the past, it is wildly believed that lung cancer drive gene mutations were mutually exclusive [30–32]. With the development of gene detection technology, cases of driver gene mutations coexistence have been detected. In a study of 5125 Chinese NSCLC patients, 160 multiple genetic mutations were found including EGFR+PIK3CA, EGFR+KRAS, KRAS+PIK3CA, EGFR+BRAF, PIK3CA + BRAF, and EGFR+KRAS +PIK3CA [18]. In our cohort of 14 patients with multiple gene mutations coexistence, 12 patients were detected with EGFR mutations, and the remaining two cases were PIK3CA + KRAS/HER2 mutation (Table 5). EGFR+PIK3CA and EGFR+PTEN were the most common forms of coexistence, accounting for 28.57% (4/14) and 21.43% (3/14), respectively, and we also found 1 case of EGFR+KRAS coexistence. These results indicated that downstream pathways engaged by EGFR can be activated by certain genomic changes.

In patients with EGFR mutation, we found an adverse effect of a concomitant mutation on prognosis. The median OS to TKIs had higher trends in exclusively EGFR mutation cases when compared to coexisting mutations with EGFR tumors (*p* > 0.05 without statistical significance). Of the 9 patients with complete follow-up data, coexisting genes in most patients were PIK3CA and PTEN (5 PIK3CA + EGFR and 3 PTEN+EGFR). PIK3CA encodes PI3Ks of the IA class activated by growth factor receptor tyrosine kinases [33]. Aberrant activation of PI3K/AKT/mTOR pathway is one of the mechanisms of acquired resistance to EGFR-TK inhibitors in patients with adenocarcinoma carrying EGFR activating mutations [34]. In gefitinib-sensitive lung cancer cells with EGFR mutations and amplifications, continued activation of PI3K signaling by the PIK3CA oncogenic mutant was sufficient to abrogate gefitinib-induced apoptosis [35]. Shorter median survival was reported in patients with concomitant PIK3CA and EGFR mutations, suggesting that the presence of PIK3CA mutations may be a predictor of poor prognosis in patients with EGFR mutations [36]. Guibert et al. found patients with EGFR/PIK3CA mutations experienced worse PFS than did patients with only EGFR mutations [37]. PTEN used to be believed as a classic tumor suppressor, low expression of PTEN protein due to gene mutation or missing may excessively activate PIK3CA/AKT signal pathway and drive the process of development and metastasis of tumor [38], which related to poor prognosis of nonsmall cell lung cancer and TKIs resistance [39, 40]. For NSCLC patients with EGFR-sensitive mutations, patients with concurrent PTEN deletion mutation had a worse prognosis after TKI treatment than those with complete PTEN [41]. It has been shown that PTEN deletion and low PTEN protein expression were predictors of poor outcome in patients treated with EGFR-TKIS [39]. In our study, two patients with PIK3CA + KRAS/HER2 mutations were lost to follow-up and therefore no prognostic data were available. In a previous small cohort study, there was a shorter median survival in patients with a coexisting mutation (EGFR, KRAS, BRAF, and ALK) versus those with mutations in PIK3CA alone [29].

This is a descriptive study that is aimed at describing the genetic variations of advanced Chinese lung adenocarcinoma patients. Our data show a panoramagram of mutation pattern in Chinese stage IV lung adenocarcinoma patients. 31.58% of patients harbored multiple mutations in our cohort, which are often related to TKI resistance and poor prognosis, so whole-genome sequencing is an effective method for making appropriate treatment choices. NGS ctDNA analysis could detect genomic mutations in NSCLC patients efficiently, especially when tumor progression occurs and positive treatment adjustments need to be made. Although not all patients received 425 gene panel detection, several unknown mutations were identified which were potential targets for TKI therapy. We detected extensive sequencing in the real-world cohort, but the limitation was the small sample size, and further large sample studies are needed to confirm these findings.

## Figures and Tables

**Figure 1:** Mutation of common driver genes.

**Figure 2:** Overall survival (OS) in the presence of exclusively EGFR mutation cases compared to coexisting mutations with EGFR patients: OS = 21.0 vs. 16.0 months, *p* = 0.104.

**Table 1:** Demographic characteristic of patients.

	EGFR		*p*	ALK		*p*	PIK3CA		*p*	KRAS		*p*
	+	—		+	—		+	—		+	—	
Gender												
Male	34	46	0.354	6	74	0.895	6	74	0.877	6	74	0.877
Female	36	36		5	67		4	68		4	68	
Age (years)												
*N* < 60	35	35	0.174	6	61	0.681	5	62	0.952	3	64	0.550
*N* ≥ 60	32	50		5	80		5	80		7	78	

**Table 2:** The relationship between EGFR mutation status and patients' characteristics.

	EGFR (-)	Exclusively EGFR mutations	EGFR +coexistent mutations	*p* value
Gender				0.252
Male	36	32	5	
Female	46	26	8	
Age (years)				0.448
*N* < 60	32	28	4	
*N* ≥ 60	50	30	8	

**Table 3:** Single mutation of EGFR gene.

EGFR gene mutations	Number of patients	Percentage (%)
Exon-19 del	15	51.72
Exon-21 L858R	10	34.48
Exon-19 ins	1	3.45
Exon-20 ins	1	3.45
Exon-21 L861Q	1	3.45
Gene amplification	1	3.45
Total analyzed	29	100.00

In our cohort, exon-19 (62.16%) was the most common EGFR gene mutation, followed by exon-21 L858R mutation (27.02%).

**Table 4:** Specific distribution of common gene mutations except for EGFR mutations.

Gene	Mutation	Number	Percentage (%)
ALK	EML4-ALK	8	5.26
	D1311E	1	0.66
	K1101N	1	0.66
	NT5C1B/MIR4757 break and rearrangement	1	0.66

PIK3CA	E545K	6	3.95
	H1047L	1	0.66
	P449L	1	0.66
	M1043I	1	0.66
	Q546K	1	0.66

KRAS	G12C	5	3.29
	G13D	2	1.32
	G12A	1	0.66
	G12D	1	0.66
	G12V	1	0.66

PTEN	S59X	1	0.66
	A126T	1	0.66
	R130X truncation	1	0.66
	V317	1	0.66
	A126T	1	0.66
	L247	1	0.66

HER2	Exon-20 insertion	2	1.32
	R143Q	1	0.66

MET	Amplification	3	1.97

NF1	W2317X truncation+Y489C	1	0.66
	S436fs	1	0.66

BRAF	V600E	2	1.32

ROS-1	ROS1-CD47 fusion	1	0.66

Total		50	32.9

**Table 5:** Combinations of multiple gene coexistence mutations.

Mutation 1	Mutation 2	Mutation 3	Mutation 4	Number
EGFR 19 del	EGFR A750P			1
EGFR 19 del	EGFR E922V			1
EGFR 19 del	EGFR T790M			6
EGFR 19 del	EGFR T790M	EGFR gene amplification		1
EGFR 19 del	EGFR T790M	EGFR C797S		1
EGFR 19 del	EGFR gene amplification			3
EGFR 19 del	EGFR R689W			1
EGFR 19 del	EGFR S752			1
EGFR 20ins	EGFR~IGFBP3&LOC7 confusion	EGFR gene amplification		1
EGFR 20ins	EGFR V774			1
EGFR 21L858R	EGFR T790M			5
EGFR 21L858R	EGFR E790K			1
EGFR 21L858R	EGFR T790M	EGFR L62R		1
EGFR 21L858R	EGFR T790M	EGFR T725M	EGFR gene amplification	1
EGFR 21L885R	EGFR gene amplification			2
EGFR 21L858R	EGFR L62R			1
EGFR 21L858R	EGFR L833V			1
EGFR 19 del	PIK3CA E542K			1
EGFR 19 del	PIK3CA E545K			1
EGFR 19 del	PIK3CA E545K	EGFR T790M	EGFR C797S	1
EGFR 19 del	PIK3CA M1043	PTEN S59X	EGFR T790M	1
EGFR 21 L858R	PIK3CA E545K			1
EGFR 19 del	PTEN A126T			1
EGFR 19 del	PTEN L247fs	EGFR T790M		1
EGFR 19 del	HER2 gene amplification	EGFR gene amplification		1
EGFR 19 del	KRAS G13D			1
HER2 p.771insAYVM	PIK3CA P449L			1
KRAS G12C	PIK3C A H1047L			1
EGFR 19 del	NF1 S436fs			1
EGFR 19 del	HER2 R143Q			1
EGFR 19 del	MET gene amplification	EGFR E922V		1
Total				43

**Table 6:** 13 patients were detected with unknown mutations.

Case	Mutation 1	Mutation 2	Mutation 3	Mutation 4	Mutation
1	RNF43 fusion				
2	AKT2 P24S	GNA11 R114Q	RB1 I181V	BRIP1 M1V	
3	MYC S154L				
4	AXL-IGR fusion	SP0P L149I	TP53 P98Lfs		
5	SMAD4 D424N				
6	DNMT3A H873R				
7	NRAS D47H				
8	SMO G177C				
9	APC I224M				
10	CBL E693V	FLT3 W196C	KDR N580D	NF2 A164V	
11	GNAS R632C	IKBKE F224V			
12	ATRX S1153L	EPHA3 fusion			
13	PRKCI E559X truncation	TGFBR2 G399R	INPP4B Q811E		

## Data Availability

The [population characteristics and gene sequencing] data used to support the findings of this study are included within the article.
